# Clinical Efficacy of Sanfeng Tongqiao Diwan in the Treatment of Allergic Rhinitis: A Randomized Controlled Trial

**DOI:** 10.1155/2022/2916223

**Published:** 2022-06-25

**Authors:** Jing Ma, Jiaying Luo, Zhangkai J. Cheng, Gui Chen, Zhiman Liang, Baoqing Sun, Feng Wang

**Affiliations:** State Key Laboratory of Respiratory Disease, First Affiliated Hospital of Guangzhou Medical University, Guangzhou 510120, China

## Abstract

**Objective:**

To explore the clinical effect of Sanfeng Tongqiao Diwan in the treatment of allergic rhinitis.

**Methods:**

Allergic rhinitis patients included in this study were randomly divided into control group and study group for 7 days of treatment. The control group was treated with Tongqiao Biyan Pian, while the study group was treated with Sanfeng Tongqiao Diwan.

**Results:**

After 7 days of treatment, the total effective rate of Sanfeng Tongqiao Diwan was 75.76%, which was higher than that of Tongqiao Biyan Pian (65.62%). The scores of visual analogue scale (VAS), symptom relief, Rhinoconjunctivitis Quality of Life Questionnaire (RQLQ), and Epworth sleepiness scale (ESS) in both groups were significantly improved before and after treatment (*P* < 0.05), and the improvement was most significant 24 hours after treatment. The adverse reactions in both groups were low.

**Conclusion:**

Sanfeng Tongqiao Diwan can significantly alleviate the symptoms and improve the quality of life of patients with allergic rhinitis, with less adverse reactions.

## 1. Introduction

Allergic rhinitis (AR) is characterized by seasonal or perennial nasal itching, sneezing, runny nose, congestion of nasal mucosa, and conjunctivitis sometimes caused by pollen or other allergens. AR is a common respiratory disease that usually lasts a lifetime. With the development of industry and the accompanying environmental problems, the incidence of allergic rhinitis in adults and children has reached 17.6%, causing a social and economic burden that cannot be ignored [1]. In addition, AR interferes with patients' sleep and imposes a great mental and economic burden on patients [2]. Therefore, effective solutions must be adopted to curb this rising trend.

Visual analogue scale (VAS) is a quick and simple method for evaluating the severity of AR [3] and has been widely used as an observation index in clinical trials. RQLQ can better assess the life quality of patients with allergic rhinitis [4]. ESS was used to observe the changes of lethargy [5].

Common treatments for AR include allergen avoidance, drug therapy, and allergen specific immunotherapy [6]. Although allergen avoidance is the basic treatment for most AR patients, it cannot relieve allergic symptoms [7]. Medications have been shown to be effective in managing allergy symptoms. First-line drugs for AR include antihistamines and glucocorticoids, but some drugs cause adverse effects and even toxicity [8, 9]. Previous study has demonstrated that traditional Chinese medicine (TCM) therapy can significantly improve the symptoms of allergic rhinitis and modulate the patient's immune response with fewer adverse reactions [8]. As a medicine for allergic rhinitis, Tongqiao Biyan Pian has been widely used in clinical practice and its effectiveness has been proved [10]. Tongqiao Biyan Pian is mainly composed of Astragalus membranaceus, Atractylodes, Fangfeng, Asarum, Xanthii, etc., while the main components of Sanfeng Tongqiao Diwan are Scutellaria baicalensis, Schizonepeta schizonepeta, Asarum, and Qianghuo. The main ingredients of these two drugs both have anti-inflammatory and antiallergic effects [11–13]. In addition, Sanfeng Tongqiao Dripping pills are also extracted by steam distillation of volatile oil, which does not contain the toxic ingredient aristolochic acid, and its efficacy has been verified in animal models of allergic rhinitis [14, 15]. Therefore, in this study, 65 patients with allergic rhinitis were selected to observe the improvement of clinical symptoms and quality of life after taking with Sanfeng Tongqiao Diwan.

## 2. Materials and Methods

### 2.1. Participants

From September 2020 to March 2021, 65 patients with allergic rhinitis were selected from the outpatient department of the First Affiliated Hospital of Guangzhou Medical University. The protocol of this study was reviewed and approved by the Ethics Committee of the Research Project of the First Affiliated Hospital of Guangzhou Medical University (YRRY 2020 No. 100), and all patients signed the informed consent.

The inclusion criteria were as follows: (1) 18-70 years of age. (2) It met the requirements of the Chinese guideline for diagnosis and treatment of allergic rhinitis (2022, revision) [16] and the Guideline for Clinical Trials of New Patent Chinese Medicines [17], and the allergic rhinitis was in the acute attack stage. The exclusion criteria were as follows: (1) pregnant and nursing women; (2) serious infection occurs in medical records, and the infection was uncontrolled; (3) patients who took H1-antihistamines, corticosteroids, and other drugs orally within 7 days; (4) personnel who are taking part in other clinical trials; and (5) lack of behavior and cognitive ability to understand the content of informed consent form.

### 2.2. Randomization

Patients who met the eligibility criteria and signed informed consent forms were randomly assigned to either the study or the control group. Envelop method was adopted for randomization, in which the random grouping scheme of research objects was stored in a sealed envelope. The Chinese red envelopes were opened in the order in which the patients were enrolled, and each patient was assigned to a group based on the allocation scheme inside the envelope.

### 2.3. Procedure

This study was a nonblind, randomized, controlled study in which Sanfeng Tongqiao Diwan was used as the study group and Tongqiao Biyan Pian as the control group. According to the instructions, patients in the study group were given Sanfeng Tongqiao Diwan (20 pills each time), 3 times a day, and the control group was given Tongqiao Biyan Pian, 6 tablets each time, 3 times a day. The whole course of treatment was seven days.

Sixty-five patients enrolled in this study completed the entire treatment process without shedding. All patients underwent security inspection and allergen skin prick test before enrollment and were enrolled after doctor's review. We will instruct the patients to fill out the questionnaire (VAS, RQLQ, ESS, and the symptom relief questionnaire) by telephone 24 hours and 4 days after medication. On the 7^th^ day of return visit, the remaining drugs will be recovered and the security inspection and questionnaire return will be conducted again (Figure 1).

### 2.4. Outcome Measures

VAS was used to score the symptoms of nasal congestion, runny nose, hypoolfaction, and so on in the two groups, and each symptom has a minimum score of 0 and a maximum score of 10. RQLQ was used to score the patients' sleep, activity, actual problems, nasal symptoms, ocular symptoms, nonnasal-ocular symptoms, and emotions, with 0~6 points for each item. ESS was used to observe the changes of drowsiness after taking Sanfeng Tongqiao Diwan. The symptom relief questionnaire was used to evaluate the clinical symptom relief rates of patients with allergic rhinitis treated with Sanfeng Tongqiao Diwan at 24 h, 4 d, and 7 d after medication.

According to nimodipine method, the total curative effect of TCM (traditional Chinese medicine) syndromes was measured. Efficacy index = (scores before treatment − scores after treatment)/scores before treatment × 100%. Cure: the clinical symptoms and signs of TCM disappeared completely or basically, and the symptom score decreased by not less than 90 points. Remarkable effect: the clinical symptoms and signs of TCM were obviously improved, and the symptom score decreased by not less than 70 points. Effective: the clinical symptoms and signs of TCM were improved, and the score of syndrome score was reduced by 30 points or more. Ineffective: the clinical symptoms and signs of TCM have not improved significantly, and the symptom scores have decreased by less than 30 points. The symptoms and signs, blood routine, urine routine, liver, and kidney series tests were performed before and after treatment.

### 2.5. Statistical Analysis

The SPSS 20.0 software was used to make statistical description and analysis. Qualitative data were expressed by rate or constituent ratio, and statistical analysis was performed by chi-square test. The quantitative data are described with mean standard deviation, statistical analysis by *T* test, and bilateral test, and two-sided *P* value less than 0.05 indicated statistically significant.

## 3. Results

### 3.1. Patient Characteristics

The study group consisted of 33 cases, 19 males and 14 females, and the average age was 30.39 ± 1.67 years old. The control group consisted of 32 cases, 17 males and 15 females, and the average age was 30.68 ± 2.08 years old. For all baseline data, there was no significant difference between the two groups (Table 1).

### 3.2. Compare the VAS, Symptom Relief, RQLQ, and ESS Scores before and after Treatment between the Two Groups

There was no significant difference between the two groups in VAS, symptom relief, RQLQ, and ESS scores before and 7 days after treatment (Table 2). However, the compliance, symptom relief questionnaire, VAS, RQLQ, and ESS scores of the patients in the study group were improved significantly after seven days of treatment. But there was no significant difference in the improvement of the ESS score before and after treatment in the control group (Table 2).

From the volcano map, we found that the VAS, symptom relief, RQLQ, and ESS scores of the study group were significantly improved before and after the treatment (Figure 2 and Table 2), and all scores related to nasal symptoms improved significantly (Figure 2), such as VAS (nasal congestion 1 and runny nose), symptom relief (nasal congestion 2, runny nose, and congestion of nasal mucosa), and RQLQ (nasal symptoms). In addition, we found changes in the levels of total protein and albumin in liver function, but these changes were not clinically significant.

### 3.3. Changes of the Questionnaire Scores in the Two Groups during Treatment

We analyzed the VAS, symptom response, RQLQ, and ESS scores of the two groups of patients with allergic rhinitis after 24 hours, 4 days, and 7 days of treatment. After research, we found that the scores of all questionnaire showed a downward trend (symptoms improvement). In our analysis, we found that after 24 hours of treatment, the symptom improvement of allergic rhinitis patients was the most significant (Figure 3).

### 3.4. Comparison of Clinical Efficacy of the Two Groups

The total effective rate of the study group was higher than that of the control group, but there was no significant difference in the clinical improvement between the two groups after 7 days of treatment (*P* > 0.05, Table 3).

### 3.5. Comparison of Adverse Reactions between the Two Groups

Adverse reactions of the two groups before and after treatment were palpitation, headache, and gastrointestinal discomfort. There was no significant difference between the two groups in the incidence of adverse events (*P* > 0.05, Table 4).

## 4. Discussion

Allergic rhinitis belongs to the category of “allergic rhinitis” in traditional Chinese medicine. Its clinical manifestations are nose and eye symptoms, which seriously affects the quality of life. Theoretically speaking, the pathogenesis of this disease is deficiency of lung, spleen, and kidney and lack of vital qi in the body, which is caused by wind and cold invading nasal orifices. The choice of treatment for AR patients depends on several factors, including the severity of symptoms, age, patient preference, patient compliance, and cost [18]. Chinese medicine, as a new drug therapy, has remarkable curative effect on improving the symptoms of allergic rhinitis and the immune status of patients [19].

This study was a single-center, open-label, and randomized controlled trial. The results showed that after seven days of administration, the overall effective rate of Sanfeng Tongqiao Diwan on allergic rhinitis is 75.76%, which was higher than that of Tongqiao Biyan Pian (65.62%). In VAS, RQLQ scores, and clinical improvement, there was no statistical difference between Sanfeng Tongqiao Diwan and Tongqiao Biyan Tablet (*P* > 0.05), but the symptoms of the patients improved obviously after treatment (*P* < 0.05). Further analysis of the whole treatment process showed that after 24 hours of administration, all symptoms improved significantly. In terms of safety, the adverse reactions of the two groups after treatment were low, with no significant difference (*P* > 0.05).

It is well known that the treatment of allergic rhinitis patients is mainly symptomatic treatment, and symptom control has become the main goal of treatment. Up to now, there is no way to cure this disease. A recent study in Taiwan Province showed that as high as 30-50% of allergic patients use traditional Chinese medicine to treat the disease, and the hospitalization rate was lower than that of patients only treated with western medicine [20]. Another recent meta-analysis on the treatment of allergic rhinitis with traditional Chinese medicine involved 11 RCT studies and more than 300 patients and concluded that CHM might significantly improve the life quality of allergic rhinitis [21], which coincides with our study. Among them, some traditional Chinese medicine preparations for the treatment of allergic rhinitis have been widely evaluated, the efficacy of Jade Screen [22] is comparable to that of receptor impedance agent, and Xinyi San [23] has a significant effect in alleviating nasal symptoms.

Sanfeng Tongqiao Diwan is a prescription summarized by famous physicians in China through practice for the treatment of acute nasal inflammation and acute attack of chronic nasal inflammation. It consists of four components, namely, Scutellaria Baicalensis, Schizonepeta, Asarum, and Qianghuo. Scutellaria [12] can reduce the infiltration of mast cells, eosinophils, and goblet cells by regulating the systemic immune response of Th cells by regulating B cells, thus reducing the production of allergic mediators and alleviating the symptoms of AR [13]. Schizonepeta and Qianghuo have anti-inflammatory effects [24–26]. At present, Sanfeng Tongqiao Diwan has been approved for marketing to improve and relieve symptoms such as nasal congestion, runny nose, sneezing, nasal congestion, and so on [27, 28].

As a major global issue, the pathogenesis and molecular mechanism of AR are still unclear. The etiology of AR is influenced by many factors, such as heredity and environment. The nature of the disease determines that this problem is a common cross-disciplinary problem. In this study, the pathogenesis and treatment of rhinitis were combined, and a comparative study of the two schemes and bioinformatics statistical analysis were carried out. The results showed that Sanfeng Tongqiao Diwan played a significant role in improving the clinical symptoms and quality of life, further supporting the theoretical feasibility of traditional Chinese medicine and the effectiveness of the drugs, and providing an effective basis for new treatment and a breakthrough point for drugs in the future.

Although Chinese medicine has been widely used for the treatment of allergic diseases, it seems that there is still a lack of conclusive evidence to determine the effectiveness of Chinese medicine for allergic diseases according to the current published data [29]. In this study, we found that the effective rate of the Sanfeng Tongqiao Diwan group was higher, but due to the limitation of sample size, no statistical difference was found in the improvement of symptoms between the two groups. Therefore, we will conduct a larger randomized controlled trial with a longer duration to confirm the efficacy of Sanfeng Tongqiao Diwan on allergic rhinitis.

## 5. Conclusions

To sum up, Sanfeng Tongqiao Diwan can significantly improve the clinical symptoms and quality of life of patients with AR attack, and it is safe.

## Figures and Tables

**Figure 1:** Study design.

**Figure 2:** Volcanic map.

**Figure 3:** Changes of patients' questionnaire score in different periods. The solid line was the study group, and the dashed line was the control group.

**Table 1:** Baseline characteristics of patients.

	Sanfeng Tongqiao Diwan (*n* = 33)	Tongqiao Biyan Pian (*n* = 32)	*P*
Age (mean ± SD)	30.39 ± 1.67	30.68 ± 2.08	>0.05
Gender (male/female)	19/14	17/15	
Course of the disease (mean ± SD)	10.96 ± 1.18	11.96 ± 1.36	
Compliance (%)	0.96 ± 0.10	0.97 ± 0.10	
Total VAS score	17.52 ± 1.42	17.00 ± 1.46	
Total symptom relief score	20.15 ± 0.68	19.4 ± 0.75	
Total RQLQ score	2.42 ± 0.17	2.52 ± 0.16	
Activity limitation	2.62 ± 0.22	2.85 ± 0.20	
Sleep problems	1.94 ± 0.22	1.84 ± 0.25	
Nonnose/eye symptoms	2.16 ± 0.20	2.09 ± 0.16	
Practical problems	3.78 ± 0.24	3.69 ± 0.23	
Nose symptoms	2.86 ± 0.22	3.38 ± 0.22	
Eye symptoms	1.61 ± 0.21	1.82 ± 0.25	
Emotion	1.97 ± 0.22	1.96 ± 0.25	
ESS score	6.54 ± 0.64	5.66 ± 0.59	

*P* value was a bilateral significance test, and *P* < 0.05 was considered statistically significant.

**Table 2:** Changes of questionnaire scores before and after treatment in two groups.

	Study (*n* = 33)			Control (*n* = 32)		
	Before therapy	After therapy	*P*	Before therapy	After therapy	*P*
Compliance (%)	0.96 ± 0.10			0.97 ± 0.10		<0.001
Total VAS score	17.52 ± 1.42	8.30 ± 1.08	<0.001	17.00 ± 1.46	8.20 ± 1.06	<0.001
Total symptom relief score	20.15 ± 0.68	12.06 ± 0.70	<0.001	19.4 ± 0.75	11.84 ± 0.89	<0.001
Total RQLQ score	2.42 ± 0.17	1.29 ± 0.14	<0.001	2.52 ± 0.16	1.29 ± 0.16	<0.001
Activity limitation	2.62 ± 0.22	1.54 ± 0.19	<0.001	2.85 ± 0.20	1.59 ± 0.20	<0.001
Sleep problems	1.94 ± 0.22	0.83 ± 0.15	<0.001	1.84 ± 0.25	0.89 ± 0.17	0.004
Nonnose/eye symptoms	2.16 ± 0.20	0.95 ± 0.12	<0.001	2.09 ± 0.16	1.07 ± 0.14	<0.001
Practical problems	3.78 ± 0.24	1.90 ± 0.18	<0.001	3.69 ± 0.23	1.89 ± 0.21	<0.001
Nose symptoms	2.86 ± 0.22	1.80 ± 0.18	0.001	3.38 ± 0.22	1.68 ± 0.21	<0.001
Eye symptoms	1.61 ± 0.21	0.95 ± 0.15	0.022	1.82 ± 0.25	0.76 ± 0.16	0.001
Emotion	1.97 ± 0.22	1.04 ± 0.18	0.002	1.96 ± 0.25	1.14 ± 0.21	0.006
ESS score	6.54 ± 0.64	4.6 ± 0.61	0.026	5.66 ± 0.59	4.66 ± 0.61	0.254

Note: VAS: visual analogue scale; RQLQ: Rhinoconjunctivitis Quality of Life Questionnaire; ESS: Epworth sleepiness scale.

**Table 3:** Changes of efficacy before and after treatment in two groups.

Group	Number of cases	Ineffective	Effective	Remarkable effect	*P*	Total effective rate
Study	33	8	23	2	0.642	75.76%
Control	32	11	17	4		65.62%

**Table 4:** Incidence rate of adverse reactions in two groups.

Group	Number of cases	Adverse reactions	Normal	*P*
Study	33	2 (6.06%)	31 (93.94%)	0.512
Control	32	1 (3.12%)	31 (96.88%)	

## Data Availability

We declare that all data was provided in our manuscript.
